RETRACTED

# microRNA-125b inhibits cell migration and invasion by targeting matrix metallopeptidase 13 in bladder cancer

**DOI:** 10.3892/ol.2013.1123

**Published:** 2013-01-10

**Authors:** DEYAO WU, JINGJING DING, LINMAO WANG, HUIXING PAN, ZHENGDONG ZHOU, JIAN ZHOU, PING QU

**Affiliations:** 1 Department of Urology, The Fourth Affiliated Hospital of Nantong Medical College, Yancheng City No. 1 People’s Hospital, Yancheng 224001;; 2 School of Basic Medical Science, Nanjing Medical University, Manjing 210029;; 3 Department of Thoracic Surgery, The Fourth Affiliated Hospital of Nantong Medical College, Yancheng City No. 1 People’s Hospital, Yancheng 224001, P.R. China

**Keywords:** bladder cancer, MMP13, miR-125b

## Abstract

The expression of microRNA-125b (miR-125b) has been investigated in many human cancers. It has been demonstrated to be downregulated in certain types of cancer, such as bladder cancer, thyroid anaplastic carcinomas, squamous cell carcinoma of the tongue, hepatocellular carcinoma, ovarian and breast cancer. In the present study, we examined the effects of miR-125b on bladder cancer cell migration and invasion. Following transfection of miR-125b, the expression of miR-125b was analyzed in T24 and EJ bladder cancer cells. Additionally, cell migration, cell invasion and luciferase assays, as well as western blot analysis were conducted in the bladder cancer cells. In this study, we demonstrated that miR-125b inhibited cell migration and invasion in T24 and EJ cells. We also provided the first evidence that miR-125b may directly target matrix metalloproteinase 13 (MMP13) in bladder cancer. Our study provided evidence that miR-125b suppresses cell migration and invasion by targeting MMP13 in bladder cancer cell lines. These results suggested that miR-125b could be used for the development of new molecular markers and therapeutic approaches to inhibit bladder cancer metastasis.

## Introduction

Bladder cancer is one of the most common malignancies worldwide. In the western world it is the seventh most common malignancy among males, following lung, prostate, colon, stomach, liver and esophageal cancer. In addition, bladder cancer represents the second most common cause of mortality among individuals with genitourinary tumors. It was estimated that there would be 70,530 new cases and 14,680 deaths due to bladder cancer in 2010 (1–3). Bladder cancer is comprised of tumors that exhibit a wide spectrum of clinical behavior. Approximately 90% of patients with bladder cancer have transitional cell carcinoma (TCC), whereas 5% exhibit squamous cell carcinomas and 1–2% have adenocarcinomas (3,4). Currently, there are many therapeutic modalities available for use depending on the extent of the disease. The treatment methods include surgery, intravesical chemotherapy, radiation therapy and systemic chemotherapy (5). The majority (50–80%) of patients with superficial TCC who solely undergo transurethral resection of bladder (TURB) suffer from recurrence. In 16–25% of these cases, superficial tumors recur with a higher grade, mostly within the first year following TURB (6). Therefore, for an improved prognosis, new therapeutic targets and approaches should be sought in order to suppress cancer recurrence.

microRNA (miRNA) belongs to a class of endogenously expressed, non-coding small RNA and contains ∼22 nucleotides (7). miRNAs are transcribed as hairpin pri-miRNAs and processed into pre-miRNAs by Drosha, an RNAse III endonuclease complexed with DGCR8. Pre-miRNAs are exported into the cystoplasm by Exportin 5 prior to cleavage by Dicer into mature miRNAs (8). Mature miRNAs are important in cell growth, proliferation, differentiation and cell death (9–11). It has also been proposed that miRNAs regulate the expression of ∼1/3 of human genes (12,13). miRNAs regulate gene expression at the post-transcriptional level through imperfect base pairing with the 3′-untranslated regions (3′-UTR) of target mRNAs (7). A growing body of evidence indicates that miRNAs are aberrantly expressed in numerous human cancers, and they may function as oncogenes and tumor suppressors. Upregulated miRNAs in cancer may function as oncogenes by negatively regulating tumor suppressors. By contrast, downregulated miRNAs may normally function as tumor suppressor genes and inhibit cancer by regulating oncogenes (14). It has been suggested that miRNA may be a target for cancer therapy.

RETRACTED

The expression of miRNA-125b (miR-125b) has been investigated in numerous human cancers. It has been demonstrated to be downregulated in certain types of cancer, such as bladder cancer, thyroid anaplastic carcinomas, squamous cell carcinoma of the tongue, hepatocellular carcinoma, ovarian and breast cancer, functioning as a tumor suppressor (15,16). However, miR-125b was found to be upregulated in pancreatic cancer, oligodendroglial tumors, prostate cancer, myelodysplastic syndromes and acute myeloid leukemia (17,18). In this study, we demonstrated that miR-125b was capable of inhibiting bladder cancer cell migration and invasion by targeting matrix metalloproteinase 13 (MMP13). These results enhance our understanding of the mechanisms of metastases, thus aiding the identification of new targets that may be used for the development of novel molecular markers and therapeutic approaches to inhibit bladder cancer metastasis.

## Material and methods

### Cells and culture conditions

The human bladder cancer cell lines T24 and EJ were obtained from the Shanghai Institute of Cell Biology, Chinese Academy of Sciences. The cells were cultured in Roswell Park Memorial Institute (RPMI)-1640 medium supplemented with 10% heat-inactivated fetal bovine serum, 100 U/ml penicillin and 100 mg/l streptomycin, at 37°C in a humidified atmosphere containing 5% CO_2_. Cells were subcultured every 2 days using trypsin/ethylenedinitrilotetraacetic acid (EDTA) solution (saline containing 0.05% trypsin, 0.01 M sodium phosphate and 0.53 *μ*M EDTA; pH 7.4). The study was approved by the faculty/institutional research committee of Yancheng City No. 1 People’s Hospital, Yancheng, China.

RETRACTED

### Quantitative reverse transcription-polymerase chain reaction (RT-PCR) for miR-125b after transfection with miR-125b mimics

Total RNA was extracted from cells using TRIzol reagent (Invitrogen Life Technologies; Carlsbad, CA, USA). Real-time qRT-PCR for miR-125b was performed with SYBR-Green miRNA assay (Genepharma; Shanghai, China) according to the manufacturer’s instructions. The primer sequences for miR-125b were as follows: Forward: ACTGATAAATCCCTGAGACCCTAAC and reverse: TATGGTTGTTCTGCTCTCTGTCAC. Briefly, a total of 500 ng RNA was used for the initial reverse transcription reaction with the gene specific stem-loop RT primer available in the kit. Real-time PCR was performed in an AB7300 thermal cycler (Applied Biosystems; Foster City, CA, USA) using the miR-125b primer set and the double-stranded DNA binding dye SYBR-Green. GAPDH was used as the internal control. The primers for GAPDH were as follows: Forward: GAAATCCCATCACCATCTTCCAGG and reverse: GAGCCCCAGCCTTCTCCATG. Every sample was replicated three times with no RT or template control included. Data were analyzed by comparing the Ct values.

### Transfection of miR-125b mimics, NC and luciferase reporter plasmid

Mature miR-125b mimics and scrambled control (NC) were designed and synthesized by Genepharma. The sequence of miR-125b mimics and scrambled control are listed in Table I. The insertion fragment was confirmed by DNA sequencing. Cell transfection and co-transfection were performed using Lipofectamine 2000 (Invitrogen Life Technologies) according to the manufacturer’s instructions.

### Cell migration and invasion assay

Cell motility was measured using an 8-*μ*m-pore polycarbonate membrane Boyden chamber insert in a Transwell apparatus (Costar; Cambridge, MA, USA). The transfected cells (miR-125b mimics and NC) growing in the log phase were treated with trypsin/EDTA solution, washed once with serum-containing RPMI-1640 medium, centrifuged and re-suspended as single-cell solutions. A total of 1×10^5^ cells in 0.2 ml serum-free RPMI-1640 medium were seeded on a Transwell apparatus. RPMI-1640 containing 20% FBS (600 *μ*l) was added to the lower chamber. An invasion assay was conducted following the same procedure, with the exception that the filters of the Transwell chambers were coated with 30 *μ*g Matrigel (BD Biosciences; San Jose, CA, USA). Following incubation of the cells for 12–24 h at 37°C in a 5% CO_2_ incubator, cells on the top surface of the insert were removed by wiping with a cotton swab. Cells that migrated to the bottom surface of the insert were fixed in 100% methanol for 2 min, stained in 0.5% crystal violet for 2 min, rinsed in PBS and then subjected to microscopic inspection (×200). Values for invasion and migration were obtained by counting five fields per membrane and represented the average of three independent experiments.

RETRACTED

### Luciferase assay

Firefly luciferase reporter plasmids containing 3′UTR of the MMP13 gene were obtained from SwitchGear Genomics (Menlo Park, CA, USA). The mutations were generated with the predicted target site of MMP13 3′UTR using the QuickChange XL sitedirected mutagenesis kit (Stratagene, La Jolla, CA, USA). Cells were plated in a 12-well plate at ∼90% confluence and transfected with 0.5 *μ*g reporter plasmid, 50 nmol miR-125b mimics or miR-Ctrl using Lipofectamine 2000. Each sample was also co-transfected with 0.05 *μ*g pRL-CMV plasmid expressing Renilla luciferase as an internal control for transfection efficiency. Twenty-four hours after transfection, cells were harvested with passive lysis buffer, according to the manufacturer’s instructions. Firefly luciferase activity and Renilla luciferase activity were measured with a luminometer (Tecan; Theale, UK). Firefly luciferase activity was normalized to Renilla luciferase activity for each transfected well. Each assay was replicated three times.

### Western blot analysis

Primary antibodies used in this study, including MMP13 and β-actin, were purchased from Bioworld Technology (Louis Park, MN, USA). Total protein of cells was prepared using radioimmunoprecipitation assay (RIPA) lysis buffer. Protein concentration in the resulting lysate was determined using the bicinchoninic acid protein assay. Equal amounts of protein were loaded onto a sodium dodecyl sulphate-polyacrylamide gel electrophoresis (SDS-PAGE) gel and transferred to a polyvinylidene fluoride (PVDF) membrane. Following blocking with 5% degreased milk in Tris-buffered saline and Tween-20 (TBST; containing 0.1% Tween-20), the membranes were incubated overnight with the appropriate primary antibody. Subsequently, the membranes were washed and incubated with the corresponding horse-radish peroxidase conjugated secondary antibody at 1:1000 dilution in TBST. The blot was developed with enhanced chemiluminescence (ECL) solution (Pierce; Rockford, IL, USA) and photographed by the FluorChem imaging system (Alpha Innotech; San Leandro, CA, USA). The intensity of each spot was read and analyzed with the AlphaEaseFC software. β-actin was used as the loading control.

RETRACTED

### Statistical analysis

Data were presented as mean ± standard deviation, and compared using the Student’s t-test in Stata 10.0 (StataCorp.; College Station, Texas, USA). A two-tailed P<0.05 was considered to indicate a statistically significant difference.

## Results

### Expression of miR-125b following transfection of miR-125b in T24 and EJ cells

We assessed the endogenous levels of miR-125b in T24 and EJ cells, as well as the expression following transfection of miR-125b every 24 h, as demonstrated in Fig. 1. The basal expression of miR-125b was barely detectable, and therefore not shown in Fig. 1. After transfection of miR-125b, the expression level was dramatically increased, then gradually decreased between 24 h and 144 h after transfection.

### miR-125b suppresses cell migration and invasion in T24 and EJ cells

To measure the effect of miR-125b on tumor cell migration and invasion, the Transwell apparatus assay was performed (Fig. 2). In the migration assay, we found that miR-125b groups exhibited a 47.61±8.25% decrease in cell migration in T24 cells and a 54.17±6.73% decrease in that of EJ cells, compared with the controls. In the invasion assay, we found that miR-133a groups demonstrated a 48.45±7.22% decrease in cell migration in T24 cells and a 51.17±6.34% decrease in that of EJ cells, compared with the controls. These results indicated that miR-125b reduced the migration and invasion in bladder cancer T24 and EJ cells.

### MMP13 is downregulated following the overexpression of miR-125b in T24 and EJ cells

We performed western blot analysis to investigate whether MMP13 expression was decreased following the transfection of miR-125b mimics in bladder cancer cell lines T24 and EJ. As demonstrated in Fig. 3, MMP13 was significantly downregulated in bladder cancer T24 and EJ cell lines following the overexpression of miR-125b (P<0.05). These results indicated that miR-125b reduced the protein level of MMP13 in bladder cancer cells.

### MMP13 is a direct target gene of miR-125b in bladder cancer

According to a computational prediction, there is an evolutionarily conserved putative binding site of miR-125b in MMP13 3′UTR. Luciferase reporter assays were performed to evaluate whether MMP13 is a true target of miR-125b. As demonstrated in Fig. 4, overexpression of miR-125b suppressed MMP13 3′UTR-luciferase activity by 41% in T24 cells and by 43% in EJ cells, compared with the controls (P<0.05). Mutation of four nucleotides within the seed-matching sequence of the predicted miR-125b binding site abolished the inhibitory effect of miR-125b on luciferase activity. Therefore, MMP13 may be a direct target of miR-125b *in vitro*.

RETRACTED

## Discussion

In humans, miR-125 has two mature isoforms, miR-125a and miR-125b, encoded by three distinct genes: miR-125a, miR-125b-1 and miR-125b-2. miR-125b-1 and miR-125b-2 map to 11q24.1 and 21q21.1, and their precursors are processed to form the same mature miRNA, miR125b (19). miR-125b is a well-characterized miRNA. Although dysregulation of miR-125b has been demonstrated to occur in multiple human cancer types, its role in disease is not completely understood (20), as in certain cell types it is observed to have an oncogenic role, while in others it exhibits a tumor suppressive role. For example, miR-125b expression is upregulated in prostate cancer, and it stimulates androgen-independent growth of prostate cells (21). By contrast, miR-125b is down-regulated in breast cancer, osteosarcoma and bladder cancer, and it suppresses tumor growth *in vitro* and *in vivo*(22–24). In a previous study, it was demonstrated that miR-125b was downregulated in the keratinocytes of psoriasis, which is an inflammatory skin disease characterized by non-malignant hyperproliferation of keratinocytes, and the miR-125b inhibited cell proliferation in human primary keratinocytes (25). The seemingly paradoxical findings indicate that the biological function of miR-125b is complex and highly cell-type dependent, which may result from the varied expression contexts of miR-125b target genes in each tumor.

Identification of miR-125b target genes is critical for understanding the role of miR-125b in tumorigenesis, and is important for defining novel therapeutic targets. To date, ERBB2/ERBB3, Bak1, CYP24, NR2A, TNF-a Bmf, Smo and p53 have been identified as targets of miR-125b (26). In bladder cancer, miR-125b was able to inhibit the proliferation and suppress the bladder cancer cells, to form colonies *in vitro* and to develop tumors *in vivo* by targeting E2F3 (23). In the present study, we demonstrated that miR-125b transfection resulted in decreased cell migration and invasion in bladder cancer T24 and EJ cells by targeting MMP13. It is concordant with the recent finding in human cutaneous squamous cell carcinoma (27). Our finding suggested that miR-125b may be used for the development of new molecular markers and therapeutic approaches to inhibit bladder cancer metastasis.

MMPs are a family of structurally related zinc-dependent endopeptidases, which, as a group, are capable of degrading essentially all extracellular matrix (ECM) components. There are 24 soluble and membrane-anchored members of the MMP family in humans that demonstrate extensive sequence homology and overlap, but distinct substrate specificities (28).MMPs are found in both normal and pathological tissue in which matrix remodeling is involved, including embryonic development, wound healing, arthritis and angiogenesis, as well as tumor invasion and metastasis (29,30). Therefore, elevated levels of MMPs have been detected in the serum and urine of patients with numerous different types of cancer, including cancer of the bladder, breast, lung, colon, head and neck, as well as melanoma (31). Proteolytic activity of the MMPs is regulated at several levels, most notably via gene transcription, activation via proteolysis of a propeptide, cell compartmentalization and inhibition by the endogenous tissue inhibitors of metalloproteinases (TIMPs) (32). Although they have pro-invasive properties, the functions of MMPs have been demonstrated to be significantly more widespread than simply facilitating migration and invasion. They are also involved in processes such as tumor initiation and progression, activation of chemokines and growth factors, angiogenesis and apoptosis induction. Therefore, it is not surprising that numerous MMPs have been identified in cancer tissue (33).

RETRACTED

MMP13 was first identified in breast carcinoma (34). Compared with the other MMPs, MMP13 has wide substrate specificity and a limited expression pattern (35). Physiological expression of MMP13 is observed to be limited to tissues undergoing rapid connective tissue remodeling, such as during fetal bone development, post-natal bone remodeling and gingival wound repair (36). However, MMP13 is expressed in various diseases involving degradation of collagenous ECM and in malignant tumors, such as squamous cell carcinomas of both the head and neck, and the vulva, cutaneous basal-cell carcinomas, chondrosarcomas and melanomas. In bladder cancer, it was demonstrated that MMP13 was expressed in tumor cells, particularly at the invading edges. In a previous study, it was demonstrated that there was no MMP13 expression in normal urothelium (37). This suggested that MMP13 may serve as a marker for transformation and invasion in TCC, otherwise, it may be a target for cancer therapy in order to inhibit metastasis from TCC. Our results suggested that miR-125b suppressed bladder cancer cell migration and invasion through downregulation of MMP13. This could be investigated as a predictive value for early detection of tumor recurrence and target therapy drugs to prevent bladder cancer from becoming invasive.

RETRACTED

In summary, to our knowledge, this is the first study to demonstrate that miR-125b regulates MMP13, and contributes to cell migration and invasion in bladder cancer. These findings have therapeutic implications and may be exploited for further treatment of bladder cancer. miRNA-based therapy is expected to be more efficient than the traditional single target therapy, as miRNAs regulate multiple target genes simultaneously. Thus, the likelihood of tumor cells developing resistance by accumulating mutations is smaller. Future studies are required to address whether the potential of miR-125b may be fully realized in cancer treatment. If so, this may be beneficial for the treatment of bladder cancer.

## Figures and Tables

**Figure 1:** Expression of miR-125b in T24 and EJ cells. The basal expression of miR-125b in T24 and EJ cells was barely detectable. The expression of miR-125b increased for 144 h following transfection of miR-125b. miR-125b, microRNA-125b.

**Figure 2:** miR-125b inhibition of cell migration and invasion. Representative photos and statistical plots of migration and invasion assays in bladder cancer T24 and EJ cells. Following 12 h incubation, the number of T24 and EJ cells that transversed the Transwell membrane decreased after the transfection of miR-125b, compared with the controls (Student’s t-test, P<0.05). Following 24 h of incubation, the number of T24 and EJ cells that transversed the Transwell membrane pre-coated with Matrigel also decreased after the transfection of miR-125b, compared with the controls (Student’s t-test, P<0.05). miR-125b, microRNA-125b; NC, scrambled control.

**Figure 3:** MMP13 expression significantly decreased in T24 and EJ cells following transfection of miR-125b, compared with the controls (P<0.05). MMP13, matrix metalloproteinase 13; miR-125b, microRNA-125b; NC, scrambled control.

**Figure 4:** MMP13 is a direct target of miR-125b. Luciferase activity significantly decreased following co-transfection with miR-125b and reporter plasmid in T24 and EJ cells. Overexpression of miR-125b suppressed MMP13 3′UTR-luciferase activity by 41% in T24 cells and 43% in EJ cells compared with the controls (P<0.05). Three independent experiments were performed and data are presented as mean ± standard deviation. MMP13, matrix metalloproteinase 13; miR-Ctrl, miRNA-control; miR-125, microRNA-125b.

**Table I:** Sequence of the miR-125b mimic and scrambled control.

	Sequence (5′-3′)
hsa-miR-125b	UCCCUGAGACCCUAACUUGUGA
Scrambled control	UUCUCCGAACGUGUCACGUTT

miRNA-125b, microRNA-125b.
